RETRACTED

# Soil organic carbon and labile and recalcitrant carbon fractions attributed by contrasting tillage and cropping systems in old and recent alluvial soils of subtropical eastern India

**DOI:** 10.1371/journal.pone.0259645

**Published:** 2021-12-16

**Authors:** Rakesh S., Deepranjan Sarkar, Abhas Kumar Sinha, Subhan Danish, Prateek Madhab Bhattacharya, Prabir Mukhopadhyay, Saleh H. Salmen, Mohammad Javed Ansari, Rahul Datta

**Affiliations:** 1 Department of Soil Science and Agricultural Chemistry, Uttar Banga Krishi Viswavidyalaya, Pundibari, Coochbehar, West Bengal, India; 2 Department of Soil Science and Agricultural Chemistry, Institute of Agricultural Sciences, Banaras Hindu University, Varanasi, Uttar Pradesh, India; 3 Department of Soil Science, Faculty of Agricultural Sciences and Technology, Bahauddin Zakariya University, Multan, Pakistan; 4 Department of Plant Pathology, Uttar Banga Krishi Viswavidyalaya, Pundibari, Coochbehar, West Bengal, India; 5 Department of Botany and Microbiology, College of Science, King Saud University, Riyadh, Saudi Arabia; 6 Department of Botany, Hindu College Moradabad (Mahatma Jyotiba Phule Rohilkhand University, Bareilly), Moradabad, India; 7 Department of Geology and Pedology, Faculty of Forestry and Wood Technology, Mendel University in Brno, Brno, Czech Republic; The University of Haripur, PAKISTAN

## Abstract

Conservation agriculture-based sustainable intensification (CASI) technologies comprising zero-tillage with crop residue retention (>30%) on the soil surface, diversified cropping systems, and balanced nutrient management are recognized as operative and efficacious strategies to ensure food security in the parts of South Asia. The present investigation was a component of CASI technologies undertaken in the farmers’ field of Malda (old alluvial Inceptisol) Coochbehar (recent alluvial Entisol) district, West Bengal (subtropical eastern India). This study was conducted to evaluate the short-term impact of contrasting tillage (zero and conventional) and cropping systems (rice–wheat and rice–maize) on total organic carbon (TOC) and its fractions, viz., labile pool-1 (LP1), labile pool-2 (LP2) and recalcitrant carbon (RC) fractions after 4-year trial of conservation agriculture (CA) in the old and recent alluvial soils. Soil samples were collected from three depths (0–5, 5–10, and 10–20 cm), and thus, our study was focused on two factors, viz., cropping system and tillage. Results pointed that TOC along with LP1, LP2, and RC fractions under rice–maize (RM) cropping system were significantly (*p*<0.05) greater (15–35%) over rice–wheat (RW) system as a result of higher residue biomass addition. Zero-tillage (ZT) improved the C fractions by 10–20% over conventional tillage (CT) in all aspects. TOC and its fractions were observed to be greater under the ZT system in the topmost soil depths (0–5 and 5–10 cm), but the same system failed to improve these at 10–20 cm. Interestingly, the CT increased all the fractions at 10–20 cm depth due to the incorporation of crop residues. The concentration of TOC along with its fractions decreased with increasing soil depth was evident. Comparatively, all the C fractions, including TOC were maximum in soils from Malda sites as compared to Coochbehar sites because of a higher amount of residue biomass application, higher clay content, and greater background content of C in these soils. All the studied C fractions showed a significant correlation (*r* = >0.635; *p*<0.01) with TOC among all the soil depths in both the districts but the relationship with soil texture showed some interesting results. TOC fractions were significantly correlated (*p*<0.01) with clay particles indicating that its higher stabilization with clay in old alluvial Inceptisol (Malda); while in recent alluvial Entisol (Coochbehar), sand particle showed its strong relation with TOC fractions. Higher stratification ratio (SR) in the ZT system suggested that the concentration of TOC and its fractions are confined to the upper soil layers whereas in the case of CT, by and large, the distribution of these was comparatively high in subsequent soil depths due to residue incorporation effect. The concentration of C fractions in soils followed the order: TOC > RC > LP2 > LP1. The present investigation concluded that ZT under the RM system increases the turnover rates of C in both soil types but the amount of clay influences the stabilization/storage of C.

RETRACTED

## 1. Introduction

Global warming and climate change impacts on humankind have spurred interest in enhancing atmospheric carbon dioxide (CO_2_) sequestration in the terrestrial ecosystems [1]. Human activities induced greenhouse gas (GHG) emission is the key cause for climate irregularities [2] which is severely affecting agricultural productivity [3, 4] in the form of salinity, drought, waterlogging, high temperature, toxicity, etc. [5]. About 22% of global anthropogenic GHG emissions are contributed by agriculture and its allied sectors [6]. Researchers and scientists have committed to lower GHG emissions by 40–70% compared to 2010 values [7]. Intense use of farmlands for cultivation results in loss of CO_2_ from soil to the atmosphere that decreases the soil organic matter (SOM) content [8]; while the plant activity is intimately associated with atmospheric CO_2_ [9]. SOM is made up of dead plant and animal residues, particulate organic carbon, humus carbon, and recalcitrant carbon which plays a crucial role in soil fertility, productivity, and overall quality of soil [10, 11] along with balancing environmental functions [12]. Agricultural soils act as a major sink for organic carbon (C) which helps in sequestering more C and reducing soil CO_2_ emission [13]. Connecting sustainable development goals (SDGs) to agriculture and the nutritional quality of food is one of the key tasks to raise crop productivity without compromising the sustainability of agricultural resources and environmental security through the build-up of SOM [14]. The concentration of SOM is often estimated by determining the soil organic carbon (SOC) or soil total organic carbon (TOC) content of the soil.

RETRACTED

TOC comprises several fractions or soil organic carbon pools (SOC-pools) such as labile pools and recalcitrant pools. Even a small change in the SOC-pools can significantly affect the atmospheric CO_2_ concentration [15]. The relative proportion of these pools is a reflection of the soil ecosystem including agricultural and non-agricultural soils which can directly impact the microbial activity and carbon dynamics in soil. The labile carbon fractions (LP-C) in soil are an important component that determines the soil quality and is a relatively smaller fraction of TOC having a very short half-life in soils and highly sensitive to management issues [16, 17]. Recalcitrant carbon (RC) is a larger fraction and a slow turnover rate exists in the soil system [18]. Long-term C storage is often determined by the long-lived RC fraction [19]. The chemical composition of these C pools varies with the stage of decomposition and their role in soil functioning and health [20]. Soil textural properties also play an important part in stabilising these fractions and influence the susceptibility of soil C to microbial attack [21].

Intensive tillage and improper nutrient management in the rice cropping system depletes the C pools and interrupt their dynamic [22, 23]. Any system that produces a rich source of organic material will have greater amounts of residue C. Labile C pools provide an important source of energy for soil microbes, the portion of organic matter in these pools determines how biologically fertile a soil is. Improvement in SOC profile increases the plant-available nutrients and holds enough soil moisture as these are the major components of sustainable agriculture [24]. The study of SOC fractions has been increasing interest in classifying various types or fractions of SOC such as labile and recalcitrant C with various residence or turnover times ascribed to the various fractions. These parameters also have been used as indicators for soil quality [17]. The distribution of SOC-fractions in the soil profile or stratification will help in identifying the variations in the quality of SOM of topsoil [25, 26].

RETRACTED

Tillage and residue management strongly affect the C sequestration rates, microbial activity thereby influencing the soil physicochemical and biological properties. Crop residues benefit the soil by supplying the nutrients with other co-benefits [27] and also can be used as mulch to conserve the soil moisture [28]. Thus, the addition of crop residues to agricultural soil is crucial for replenishing the annual C losses and for improving overall soil health [29, 30]. Conservation agriculture-based sustainable intensification (CASI) technologies involving minimum soil disturbance along with increased crop residue retention may hold the key to address the C losses [31]. Continuous crop rotation in agriculture management practices aid in the provision of improving soil carbon stocks [15, 23]. Zero-tillage (ZT) under CASI technology has been identified as an important practice to increase soil aggregation and C sequestration [32] as compared with conventional tillage (CT).

The present study was undertaken to assess the effect of different tillage and crop residue management practices on labile and recalcitrant C fractions using experimental fields of the Australian Centre for International Agriculture Research (ACIAR) funding project “Sustainable and Resilient Farming System Intensification” (SRFSI). The research was conducted in farmers’ fields of the ongoing ACIAR-SRFSI research project which was initiated in 2013 to demonstrate the advantages of CA systems over the conventional system across two districts [Malda, old alluvial Inceptisoland Coochbehar, recent alluvial Entisol] of West Bengal, India.

Our study hypothesized that alteration in tillage and crop management practices along with the adoption of different cropping systems will have a differential impact on the composition of labile and recalcitrant carbon fractions at varying soil depths. Therefore, in this background, objectives of the present investigation included (i) to evaluate the response of labile and recalcitrant carbon fractions to different tillage practices and cropping systems over the experimental period of 4 years, (ii) to explore the stratification of carbon fractions in the soil profiles of different agroecosystems, and (iii) to study the relationship of TOC and its fractions with soil textural properties under different agro-climatic conditions.

## 2. Materials and methods

### 2.1. Description of experimental sites

The experiment was carried out in the fields of the ACIAR-SRFSI project which was executed in two different districts, i.e., Malda [24°56′ 38′′ N 88°08′19′′ E] and Coochbehar [26°16′ 16′′ N 29°24′52′′ E], West Bengal, India. The project was implemented in 2013–14 in the field trials of farmers in 5 sites of each district with different cropping systems (Rice-Wheat and Rice-Maize) and tillage (ZT and CT). For the present study, soil sampling was done in 2017 (after 4 years of trial). Totally, four sites from Malda and three sites from Coochbehar district (discarded 1 site due to technical error) were selected (Table 1) to study the effect of different tillage and cropping systems on labile and recalcitrant carbon pools. The experimental design was a factorial completely randomized design (CRD). Soils of Malda are fine loam to coarse loam in texture with high mean TOC of 11.62 g kg^-1^, and high bulk density, neutral to alkaline belongs to old alluvial Inceptisol; while the Coochbehar soils are coarse loam in texture with mean TOC of 9.77 g kg^-1^, low bulk density, and acidic pH belongs to recent alluvial Entisol as classified under National Bureau of Soil Survey and Land Use Planning (NBSS & LUP) soil classification of West Bengal. The pH, TOC, total nitrogen (N), soil texture, and bulk density along with soil profile description of the experimental soils are given in S1 Table.

RETRACTED

**Table 1:** Details of cropping system, tillage, and sampling depths in 7 sites of 2 districts of West Bengal, India.

District	Site	Village Name	Cropping System	Tillage	Sampling Depth (cm)
Malda	1	Ugritola	Rice–Wheat & Rice–Maize	Zero & Conventional	0–5, 5–10 & 10–20
	2	Mohadipur			
	3	Bidyandapur			
	4	Gowrangapur			
Coochbehar	5	Ghugumari	Rice–Wheat & Rice–Maize	Zero & Conventional	0–5, 5–10 & 10–20
	6	Falimari			
	7	Patchara			

### 2.2. Crop management practices

Wheat and maize crops were sown immediately after the harvest of the rice crop. The sowing dates varied from the first week of November to the last week of December. An individual cropping system (RW and RM), consisted of two tillage systems (CT and ZT) was established at all 42 (each 21 for RM and RW) farmers’ fields in the seven selected field sites (FS) of Malda and Coochbehar. The area under each treatment plot was 666 m^2^ (0.07 ha). The tillage and cropping systems used for CT were: Puddled transplanted rice (PTR)–CT maize or wheat; and ZT: Unpuddled transplanted rice (UPTR)–ZT maize or wheat. Rice seedlings were transplanted at 22 cm row spacing in the ZT using a mechanical transplanter, and planted randomly by hand in the CT resulting in 28–30 hill m^-2^. Wheat was sown at 20 cm row spacing in the ZT with continuous seeding (180–200 plant m^-2^) and broadcasted in the CT. Maize was planted at 60 × 20 cm (row × plant) in both the ZT and CT resulting in 75000–80000 plants ha^-1^. Crops were fertilized at rates (kg ha^-1^) recommended for the area; rice 80–90 N, 15–20 P, 40–70 K; wheat 125–145 N, 20–25 P, 40–60 K; and maize 155–180 N, 20–25 P, 60–75 K using urea, di-ammonium phosphate (DAP) and muriate of potash (MOP) fertilizers respectively. Brief information on crop management practices is presented in the article of [33].

RETRACTED

### 2.3. Soil sampling

Soil samples were collected from all the 4 sites of Malda and 3 sites of Coochbehar comprising of two cropping systems (RM and RW) and two tillage systems (ZT and CT). Soil sampling was carried from three farmers of each cropping system and tillage at three depths, viz., 0–5, 5–10, and 10–20 cm after the harvest of wheat and maize crops. Samples from the multiple spots of each experimental plot were collected with the help of a 20 cm length core sampler ended with one composite sample of each depth by the proper mixing process. These samples were properly labelled and brought to the laboratory. The samples were then air-dried thoroughly in shade, pulverized, and sieved through a 2 mm mesh sieve (for the analysis of physicochemical properties) and 0.5 mm mesh sieve (for estimating TOC and its fractions). Samples were then kept in properly marked polythene packets, appropriately sealed, and stored for different experiments during the course of the investigation.

### 2.4 Soil analysis

#### 2.4.1. Total organic C (TOC)

A modified Walkley and Black method (Baker, 1976) was followed for the analysis of TOC in soil determined by the colorimetric method using sucrose as a standard. Briefly, one gram of soil sample was digested in the presence of 20 mL of 5% K_2_Cr_2_O_7_ and 10 mL of concentrated H_2_SO_4_. After cooling for 30 minutes, 50 mL of 0.4% BaCl_2_ was added and allowed to stand overnight. The intensity of the yellow/orange colour was read at 600 nm wavelength using a UV-visible spectrophotometer.

#### 2.4.2. Labile pool-I and Labile pool-II carbon (LP1 & LP2)

The two-step acid hydrolysis method [34] using H_2_SO_4_ as the extractant was used to determine the labile pools of carbon. In detail, 20 mL of 5 N H_2_SO_4_ was added to 0.5 g soil, and the samples were hydrolysed for 30 min at 105° C in sealed 100 ml capacity centrifuge tubes using a hot water bath. After cooling down, the hydrolysates were centrifuged at 6000 rpm for 10 minutes and recovered through decantation followed by washing with 20 mL de-ionized water and the washing added to the hydrolysate. This hydrolysate was considered as labile pool I (LP1) after filtering through Whatman no. 1 filter paper. The remaining residue was again hydrolysed with 2 mL of 26 N H_2_SO_4_ for 16 hours (overnight) at room temperature under continuous shaking. The next day, the concentration of the acid was then brought down to 2 N by dilution with de-ionized water (approx. 24–26 mL) and then the sample was hydrolysed for 3 hours at 105° C with occasional shaking. This second hydrolysate (labile pool 2-LP2) was recovered in the same manner as followed in LP1.

RETRACTED

The C content in hydrolysate was determined by [35] method. In brief, about 4 mL of hydrolysate was oxidised with 1 mL of 0.066 M K_2_Cr_2_O_7_ and 5 mL of concentrated H_2_SO_4_ at 150° C for 30 minutes. Samples after cooling, titrated against 0.033 M ferrous ammonium sulphate (FAS) with 2–3 drops of *o*-phenanthrolene indicator until the colour turned from greenish violet to brick red.

#### 2.4.3. Recalcitrant pool carbon (RC)

RC was estimated by the difference between the sum of two labile pools and TOC content obtained [20].


RC=TOC–(LP1+LP2)

#### 2.4.4. Stratification ratio (SR)

The stratification ratio of a soil property is defined as the ratio of its value at the soil surface to that at a lower depth [36]. This ratio for a C fraction for 0–10 cm depth was calculated by dividing its value at 0–5 cm to that of its 5–10 cm depth. Similarly, for 0–20 cm depth, the value of 0–5 cm depth was divided by its C concentration at 10–20 cm soil depth.

#### 2.4.5. Data analysis

A factorial completely randomized design CRD was employed to evaluate the main and interaction effect of cropping system, tillage, and depth on various carbon (C) fractions at *p*<0.05 with separation of means by least significant difference (LSD) in SPSS 17.0 software package. A Pearson correlation (r) test was performed to determine the relationship of TOC and its fractions with and soil textural properties at 0–5, 5–10, and 10–20 cm depths separately for Malda and Coochbehar, and the significant probability levels of the results were given at *p*<0.05 (*) and *p*<0.01 (**), respectively.

## 3. Results

### 3.1. Total organic carbon

The depth-wise concentration of TOC was decreased significantly (*p<*0.05) with an increase in depth (Fig 1). The TOC concentration in the soil varied from 8.37 to 18.74 g kg^-1^ at 0–5 cm, 7.95 to 15.72 g kg^-1^at 5–10 cm and 7.20 to 13.04 g kg^-1^ at 10–20 cm depths (Table 2). The site-4 of Malda showed a maximum concentration of TOC at all the soil depths and site-6 of Coochbehar recorded the least amount of TOC. The RM plots had a significantly (*p<*0.05) greater amount of TOC (15–30%) than RW in all the selected sites of Malda and Coochbehar districts (Table 2). Out of seven sites studied, levels of TOC increased significantly (10–15%) in ZT plots in comparison to CT plots in five sites. Interaction effect of cropping system (CS), tillage (T), and depth (D) on TOC and its fractions have been presented in S2–S5 Tables. The interplay of CS × D on TOC showed noticeably a significant (*p<*0.05) amount in both RW and RM systems under ZT compared to CT. However, the values of TOC were reported to be higher in the RM cropping system under ZT. In this study, 2 sites showed a non-significant effect of CS and T. In the lower depths (5–10 and 10–20 cm), CT enhanced the TOC compared to ZT but the interaction of CS and D was significant only in 2 sites. The interplay of T × D showed significance among all the sites (Fig 2). It showed that, except one or two sites, the ZT improved the overall concentration of TOC at the upper two layers (0–5 and 5–10 cm) in all the sites; whereas the CT increased the same (by 10–25%) in 10–20 cm layer. The CS × T × D recorded non-significant in most of the sites (data shown in supplementary files).

RETRACTED

**Fig 1:** Depth wise distribution of LP-1, LP-2, RC, and TOC in different sites of Coochbehar and Malda.

**Fig 2:** Effect of tillage system on TOC at different soil depths in the sites of Malda and Coochbehar.

**Table 2:** Effect of tillage, cropping system, and soil depth on TOC (g kg^-1^) in different sites of Malda and Coochbehar districts.

District		Malda				Coochbehar		
Location		Site-1	Site-2	Site-3	Site-4	Site-5	Site-6	Site-7
Cropping system (CS)	RW	10.24	11.40	10.64	14.54	12.96	6.63	12.40
	RM	9.57	13.13	13.12	17.13	13.60	9.05	12.51
SEM (±)		0.16	0.25	0.21	0.28	0.17	0.07	0.17
CD (*p*<0.05)		0.47	0.72	0.62	0.82	0.49	0.20	NS
Tillage (T)	ZT	10.67	12.76	11.29	15.73	13.24	8.74	13.49
	CT	9.15	11.76	12.48	15.93	13.32	6.94	11.43
SEM (±)		0.16	0.25	0.21	0.28	0.17	0.07	0.17
CD (*p*<0.05)		0.47	0.72	0.62	NS	NS	0.20	0.50
Depth (D)	0 to 5	12.45	14.80	15.39	18.74	15.56	8.37	14.31
	5 to 10	10.12	11.72	10.97	15.72	14.24	7.95	12.43
	10 to 20	7.15	10.27	9.29	13.04	10.04	7.20	10.64
SEM (±)		0.20	0.30	0.26	0.34	0.21	0.08	0.21
CD (*p*<0.05)		0.58	0.89	0.76	1.01	0.60	0.24	0.62
Interactions (Pr>F)								
CS * T (*p*<0.05)		0.67	NS	0.88	1.16	0.70	0.28	NS
CS * D (*p*<0.05)		0.81	NS	NS	NS	NS	0.34	NS
T * D (*p*<0.05)		0.81	1.25	1.08	1.42	0.85	0.34	0.87
CS * T * D (*p*<0.05)		1.15	NS	1.52	NS	1.21	0.48	1.23

R-W: Rice-Wheat CS; R-M: Rice-Maize CS; ZT: Zero-tillage; CT: Conventional tillage; Site-1: Ugritola; Site-2: Mohadipur; Site-3: Bidyanandapur; Site-4: Gowarangapur; Site-5:Ghugumari; Site-6: Falimari; Site-7: Patchara.

### 3.2. Labile pool 1 carbon

The percent contribution of LP1 fraction to TOC was observed to be 10.97 to 20.35% (Fig 3) which is lesser than the other studied fractions (LP2 and RC). With respect to the percent contribution to TOC, soils of Coochbehar recorded higher LP1 carbon. Depth-wise distribution of LP1 (Table 3 and Fig 1) showed decreasing pattern with increasing depth. The LP1 concentration in the soil varied from 1.63 to 2.74 g kg^-1^ at 0–5 cm, 1.13 to 2.15 g kg^-1^ at 5–10 cm and 0.48 to 1.68 g kg^-1^ at 10–20 cm depths (Table 3). The site-4 of Malda recorded higher LP1 at 0–5 cm depth but in the subsequent depths (5–10 and 10–20 cm), site-5 and site-7 of Coochbehar recorded higher LP1 to the tune of 25% at 5–10 cm and 40% at 10–20 cm depths respectively. As observed in TOC, the RM system significantly enhanced the LP1 in all the sites (Table 3). On average, 15% more LP1 concentration was observed in the RM system than RW. Adoption of ZT improved the LP1 to a greater extent, but in few sites (site 1 and 4) we noticed CT enhancing the same. The interaction effect of CS × T was significant (*p*<0.05) in all the sites of Coochbehar but non-significant in the two sites of Malda. The CS × D was observed to be significant in 6 sites and T × D was significant in 5 sites. The CS × T ×D revealed that ZT in Coochbehar enriched the LP1 in both cropping systems at 0–5 and 5–10 cm (Fig 4A and 4B). The CT system improved the same at 10–20 cm depth. We further noticed that in Malda, ZT failed to improve the LP1 in lower soil depths under both cropping systems. Comparatively, the RM system showed higher values under both tillage systems at all the soil depths in Malda and Coochbehar.

RETRACTED

**Fig 3:** Percent contribution of LP1, LP2, and RC to TOC.

**Fig 4:** Effect of R-W cropping system on LP1 carbon under ZT and CT management at 0–5, 5–10, and 10–20 cm depths. a. b. Effect of R-M cropping system on LP1 carbon under ZT and CT management at 0–5, 5–10, and 10–20 cm depths.

**Table 3:** Effect of tillage, cropping system, and soil depth on LP1 carbon (g kg^-1^) in different sites of Malda and Coochbehar districts.

District		Malda					Coochbehar		
Location		Site-1	Site-2	Site-3	Site-4		Site-5	Site-6	Site-7
Cropping system (CS)	RW	0.95	1.39	1.63	1.88		1.82	1.50	1.95
	RM	1.21	1.67	1.90	2.19		2.13	1.68	2.04
SEM (±)		0.019	0.019	0.051	0.042		0.035	0.015	0.021
CD (*p*<0.05)		0.057	0.057	0.149	0.122		0.102	0.044	0.062
Tillage (T)	ZT	1.05	1.69	1.79	1.94		2.02	1.73	2.18
	CT	1.10	1.37	1.73	2.14		1.92	1.45	1.81
SEM (±)		0.019	0.019	0.051	0.042		0.035	0.015	0.021
CD (*p*<0.05)		NS	0.057	NS	0.122		NS	0.044	0.062
Depth (D)	0 to 5	1.63	1.96	2.34	2.74		2.22	1.70	2.34
	5 to 10	1.13	1.43	1.62	2.00		2.15	1.68	1.97
	10 to 20	0.48	1.20	1.33	1.37		1.55	1.39	1.68
SEM (±)		0.024	0.024	0.062	0.051		0.043	0.018	0.026
CD (*p*<0.05)		0.069	0.070	0.183	0.149		0.126	0.054	0.076
Interactions (Pr>F)								
CS * T (*p*<0.05)		0.080	NS	0.211	NS		0.145	0.062	0.088
CS * D (*p*<0.05)		0.098	0.099	NS	0.211		0.178	0.076	0.108
T * D (*p*<0.05)		NS	0.099	0.258	NS		0.178	0.076	0.108
CS * T * D (*p*<0.05)		0.138	0.140	NS	NS		0.251	0.107	0.152

R-W: Rice-Wheat CS; R-M: Rice-Maize CS; ZT: Zero-tillage; CT: Conventional tillage; Site-1: Ugritola; Site-2: Mohadipur; Site-3: Bidyanandapur; Site-4: Gowarangapur; Site-5: Ghugumari; Site-6: Falimari; Site-7: Patchara.

RETRACTED

### 3.3. Labile pool 2 carbon

The LP2 carbon fraction contributed about 14.55 to 25.39% to TOC recorded 1.2 to 1.4 folds higher than LP1 (Fig 3). Depth-wise distribution of LP2 (Table 4 and Fig 1) showed the same pattern as noticed in LP2. The concentration of LP2 in the soil varied from 2.20 to 3.44 g kg^-1^ at 0–5 cm, 1.32 to 2.71 g kg^-1^ at 5–10 cm, and 0.77to 2.33 g kg^-1^ at 10–20 cm depths (Table 4). There was a significant (*p<*0.05) increase (12–18%) in LP2 in the RM system compared to the RW system in all the sites except in site-1 of Malda where the concentration was higher (by 15%) in RW. The effect of tillage on the status of LP2 was variable in all seven sites. A significant (*p<*0.05) increase in LP2 in ZT (5–10%) over CT was noted in five sites and in the other two sites, the trend was reversed. The interplay of CS × T showed that adoption of ZT significantly (*p<*0.05) increased the LP2 in both cropping systems but it was non-significant in three sites. On site-4 of Malda, there was an improvement of LP2 under CT in both RW and RM. The same trend of a higher amount of LP2 in CT was reported in site-5 of Coochbehar but under RW. Overall, the concentration of LP2 was found to be significantly better in ZT compared to CT in the RM cropping system. The interaction of CS × D for sites 1, 2, 4, 6, and 7 indicates that there was a significant (*p<*0.05) difference in LP2 distribution under the two-cropping systems among all the soil depths.

**Table 4:** Effect of tillage, cropping system, and soil depth on LP2 carbon (g kg^-1^) in different sites of Malda and Coochbehar districts.

District		Malda					Coochbehar		
Location		Site-1		Site-2	Site-3	Site-4	Site-5	Site-6	Site-7
Cropping system (CS)	RW	1.55		2.09	1.99	2.70	2.61	1.79	2.33
	RM	1.32		2.26	2.18	2.92	2.50	2.18	2.60
SEM (±)		0.034		0.025	0.064	0.046	0.036	0.018	0.027
CD (*p*<0.05)		0.099		0.074	0.187	0.134	0.105	0.054	0.080
Tillage (T)	ZT	1.43		2.27	2.13	2.69	2.53	2.14	2.52
	CT	1.44		2.08	2.04	2.93	2.58	1.83	2.40
SEM (±)		0.034		0.025	0.064	0.046	0.036	0.018	0.027
CD (*p*<0.05)		NS		0.074	NS	0.134	NS	0.054	0.080
Depth (D)	0 to 5	2.20		2.76	2.78	3.44	2.93	2.23	2.89
	5 to 10	1.32		2.22	2.12	2.66	2.71	1.95	2.50
	10 to 20	0.77		1.55	1.35	2.33	2.02	1.77	2.00
SEM (±)		0.041		0.031	0.078	0.056	0.044	0.022	0.033
CD (*p*<0.05)		0.122		0.091	0.229	0.164	0.129	0.066	0.098
Interactions (Pr>F)								
CS * T (*p*<0.05)		NS		0.105	NS	0.189	0.149	0.076	NS
CS * D (*p*<0.05)		0.172		0.128	NS	0.232	NS	0.093	0.138
T * D (*p*<0.05)		NS		NS	NS	NS	NS	0.093	0.138
CS * T * D (*p*<0.05)		0.243		0.182	NS	NS	NS	0.132	0.196

R-W: Rice-Wheat CS; R-M: Rice-Maize CS; ZT: Zero-tillage; CT: Conventional tillage; Site-1: Ugritola; Site-2: Mohadipur; Site-3: Bidyanandapur; Site-4: Gowarangapur; Site-5: Ghugumari; Site-6: Falimari; Site-7: Patchara.

RETRACTED

### 3.4. Recalcitrant carbon (RC)

This fraction contributed the maximum to TOC (54.31 to 74.50%). The depth-wise distribution of RC fraction (Table 5 and Fig 1) among different sites of Malda and Coochbehar showed a significant decrease in concentration with an increase in depth. The highest amount of RC fraction recorded in site-4 (12.55 g kg^-1^) followed by 10.41 g kg^-1^ (site 5) has been recorded at 0–5 cm depth. However, the site-6 (Falimari) recorded the lowest amount (4.45 g kg^-1^) of RC and the status among the studied depths (4.45, 4.32, and 4.05 g kg^-1^ at 0–5, 5–10, and 10–20 cm respectively) was also lower due to its similar trend of TOC concentration. Since this pool was calculated by summing the LP1 and LP2 carbon and subtracted from TOC provides similar variations as TOC. The mean results of RC (Table 5) with respect to different cropping systems showed a significant (*p*<0.05) higher amount of RC fraction in the RM cropping system than the RW cropping system except in site 1 and site 7 where the RW system recorded higher values of RC. The main effect of tillage failed to show a significant difference in the three sites (site 2, site 4, and site 5). However, site-4 presented the highest value of 11.10 g kg^-1^ under ZT over the CT (10.86 g kg^-1^). The least concentrations of RC, i.e., 4.88 and 3.66 g kg^-1^recorded in site-6 (Falimari) under ZT and CT systems respectively. The interplay between different tillage effects with soil depths (D x T) shown significantly (*p*<0.05) maximum values of RC under the ZT system (10–20% higher) against the CT (Fig 5). The uppermost depth (0–5 cm) has enormously enriched the RC in the case of ZT, where the concentration of the same fraction at the lowermost depth (10–20 cm) was higher under CT among all the sites except in site-1 and site-7 (Fig 5); where these two interaction effects showed greater amounts in ZT in the mentioned sites which is also reflected from the TOC concentration.

**Fig 5:** Effect of tillage system on RC at different soil depths in the sites of Malda and Coochbehar.

RETRACTED

**Table 5:** Effect of tillage, cropping system, and soil depth on RC (g kg^-1^) in different sites of Malda and Coochbehar districts.

District			Malda				Coochbehar		
Location			Site-1	Site-2	Site-3	Site-4	Site-5	Site-6	Site-7
Cropping system (CS)	RW		7.75	7.92	7.03	9.96	8.54	3.35	8.13
	RM		7.05	9.19	9.04	12.01	8.97	5.19	7.88
SEM (±)			0.16	0.24	0.21	0.30	0.19	0.07	0.17
CD (*p*<0.05)			0.47	0.71	0.61	0.89	NS	0.20	NS
Tillage (T)	ZT		8.19	8.80	7.37	11.10	8.70	4.88	8.79
	CT		6.61	8.32	8.71	10.86	8.82	3.66	7.22
SEM (±)			0.16	0.24	0.21	0.30	0.19	0.07	0.17
CD (*p*<0.05)			0.47	NS	0.61	NS	NS	0.20	0.50
Depth (D)	0 to 5		8.62	10.09	10.27	12.55	10.41	4.45	9.08
	5 to 10		7.68	8.07	7.23	11.06	9.38	4.32	7.96
	10 to 20		5.89	7.52	6.62	9.33	6.47	4.05	6.96
SEM (±)			0.20	0.30	0.26	0.37	0.23	0.08	0.21
CD (*p*<0.05)			0.58	0.87	0.75	1.09	0.67	0.24	0.61
Interactions (Pr>F)								
CS * T (*p*<0.05)			NS	NS	NS	1.26	0.77	0.28	NS
CS * D (*p*<0.05)			0.82	NS	NS	NS	NS	0.34	NS
T * D (*p*<0.05)			0.82	1.23	1.06	1.55	0.95	0.34	0.86
CS * T * D (*p*<0.05)			1.16	NS	NS	NS	1.34	NS	NS

R-W: Rice-Wheat CS; R-M: Rice-Maize CS; ZT: Zero-tillage; CT: Conventional tillage; Site-1: Ugritola; Site-2: Mohadipur; Site-3: Bidyanandapur; Site-4: Gowarangapur; Site-5:Ghugumari; Site-6: Falimari; Site-7: Patchara.

### 3.5. Relationship of labile and recalcitrant carbon fraction with TOC and soil textural properties

All the fractions showed a significantly positive relationship with TOC among all the soil depths (Table 6) of Malda and Coochbehar. The correlation of all these fractions varied widely with the soil textural properties (sand, silt, and clay). We observed similar relationship results at 0–5 and 5–10 cm depths but at the lowermost depth (10–20 cm), it was disparate. Interestingly, we noticed that all the C fractions (LP1, LP2, and RC) along with TOC showed a strong positive relationship with clay in Malda soils at all the depths but in Coochbehar, the scenario was different; it was correlated positively with sand. We further noticed a negative relationship of C fractions with silt particles in both the districts but at 10–20 cm depth, Malda showed a positive relation with silt.

**Table 6:** Relationship of LP1, LP2, and RC with TOC and soil textural properties.

			TOC	SAND	SILT	CLAY
0 to 5	Malda	LP1	0.925**	-0.208	-0.104	0.795**
		LP2	0.910**	-0.25	-0.079	0.850**
		RC	0.988**	-0.267	-0.002	0.720**
		TOC		-0.263	-0.034	0.783**
	Coochbehar	LP1	0.896**	0.353	-0.467	0.171
		LP2	0.844**	0.215	-0.381	0.424
		RC	0.996**	0.565*	-0.690**	0.081
		TOC		0.529*	-0.660**	0.121
5 to 10	Malda	LP1	0.635**	-0.097	-0.116	0.621*
		LP2	0.776**	0.121	-0.373	0.619*
		RC	0.966**	-0.456	0.26	0.751**
		TOC		-0.34	0.104	0.801**
	Coochbehar	LP1	0.653**	0.091	-0.159	0.189
		LP2	0.788**	0.283	-0.399	0.271
		RC	0.987**	0.600*	-0.674**	0.008
		TOC		0.545*	-0.631**	0.064
10 to 20	Malda	LP1	0.714**	-0.286	0.165	0.358
		LP2	0.803**	-0.752**	0.653**	0.796**
		RC	0.964**	-0.564*	0.513*	0.581*
		TOC		-0.627**	0.550*	0.661**
	Coochbehar	LP1	0.554*	0.16	-0.087	-0.083
		LP2	0.806**	0.571*	-0.479	0.017
		RC	0.991**	0.662**	-0.517*	-0.049
		TOC		0.648**	-0.506*	-0.049

Note

* and ** represent that correlation is significant at the 0.05 and 0.01 level (2-tailed) respectively.

RETRACTED

### 3.6. Stratification ratios of LP1, LP2, and RC at 0–20 cm soil depth

From the stratification ratio values of LP1, LP2, and RC at 0–10 (0-5/5-10) and 0–20 (0-5/10-20) cm depths under two tillage systems (Fig 6), it was evident that the higher stratification ratio values of C fractions recorded in case of ZT than CT in most of the sites. Comparatively, Malda soils resulted in greater ratio values than Coochbehar. The comparison between the two tillage systems revealed that the higher distribution of C fractions in the soil profile is much appropriate under the CT system because of frequent tillage and incorporation of residues during cultivation which exhibited lower stratification values compared to the ZT system.

**Fig 6:** Stratification ratios of LP1, LP2, and RC in 0–20 cm soil in the different sites of Coochbehar and Malda under tillage (ZT and CT) systems.

## 4. Discussion

We observed that RM plots significantly increased the amount of TOC as compared to RW is due to the excessive addition of carbon substrate in the former system than the latter, which naturally improved the TOC in soil. This outcome was in agreement with several researchers [20, 37, 38] who were reported that labile C and N levels were maximum in high substrate input systems and minimum in those with the low substrate. Plots under ZT showed higher TOC concentrations over CT. Similar higher TOC concentration in the ZT system was widely reported by many researchers [21, 39]. TOC decreased significantly with an increase in depth due to residue accumulation on the soil surface. The concentration of TOC and its fractions decreased with increasing soil depth and thus caused a natural stratification by residue accumulation on the soil surface [36, 40, 41]. In our study, we observed higher TOC concentration in both the cropping systems under ZT management; however, the RM system showed a pretty higher concentration over RW. The ZT with crop residue application at upper soil depth had distinctly higher SOC sequestration than CT with crop residue [42]. Higher TOC concentration was observed under ZT at the upper two layers (0–5 and 5–10 cm); whereas under CT, its concentration increased at 10–20 cm layer (Fig 2). A similar increment in SOC close to the soil surface (0–10 cm) under the ZT system was reported by [43]. SOC stocks below the old plough layer (28–40 cm) were slightly greater in full inversion tillage (FIT) than in ZT treatment [44]. A similar trend of the CT enhanced the TOC content in the lower layer (10–20 cm) by 18% over ZT was also reported by [45].

RETRACTED

On average, Coochbehar soils reported pretty higher values of LP1 compared to Malda. The ZT improved the concentration of LP1 over CT in all the sites except in site-1 which showed higher LP1 in CT plots. In site-1, there was poor germination due to the improper handling of the ZT machine during cultivation resulted in lower plant population ultimately lower residue addition. Soil depthwise status showed that the ZT resulted in higher LP1 at 0–5 cm while in CT, this was seen at 5–20 cm soil depth in both the cropping systems but only in some of the sites. Such variations in the distribution of LP1 in different locations are probably due to the differences in the amount of plant material input and the background TOC status of the soils. Stratification of LP1 at 0–5 cm was higher in the sites of Malda over Cooch Behar under both the cropping system was due to the differences in texture of both the places that we have discussed in detail under the stratification of the C fractions. The percent contribution of LP1 towards TOC in the entire soil depth of 0–20 cm observed in our study was in agreement with [46].

There was a significant increase in LP2 noted under the RM system among all the sites except in site-1 of Malda where the concentration was higher (by 15%) in RW. The performance of the wheat crop was better than the maize in this site due to the differences in the management practice. Additionally, the cultivation of the wheat crop is well known to the farmers due to which the crop management involved there is traditionally expertise. Further, the maize crop under ZT created a problem in germination due to low soil moisture. Therefore, the yield of maize suffered adversely (data not shared), and the effect of poor growth also influenced the status and distribution of the SOC pools. A trend of decrease in LP2 with an increase in depth was observed among all the sites and the rate of decrease varied due to the differences in texture and moisture in soils. A significant increase in LP2 in ZT was noted in five sites and in the other two sites, the trend was reverse may be due to the low mineralization of organic substances in these two sites. In-situ accumulation of labile C fractions under ZT is due to a decrease in the mineralization intensity of the SOM [47]. The variations in the status of LP2 due to the tillage treatment are because of the differences in residue management which resulted in a difference in the rate of decomposition of residues. Enriched labile C fraction is a passive pool of SOM and is not derived from microbes or sensitive to cultivation [48]. The association of LP2 with the other fractions was more distinct in soils of Malda where the effect of clay on the distribution and the status of these pools was very evident from the significant and positive correlation (Table 7) of the C fractions with clay. In contrast to this, in lighter textured soils of Coochbehar, this (C) association was more evident with sand particles and therefore, C was unstable in these soils. The chemical oxidation method of [34] also indicates the biochemical quality of the SOM. Carbohydrates of LP2 correspond to cellulose, while the LP1 include polysaccharides of both microbial origin (microbial cell walls) and plant origin (hemicelluloses, starch residues); thus, the LP II/(LP I + LP II) ratio is equivalent to the cellulose-to-total-carbohydrates ratio (Table 7). In the present study, the cellulose content (LP2) was relatively higher in the organic residues added in the soil and the residues were relatively new in origin. [34] in their study reported that as decomposition proceeds, the ratio of cellulose to total carbohydrates decreases and hence a high cellulose/total carbohydrates ratio indicated a relevant presence of fresh plant contributions.

RETRACTED

**Table 7:** LP 2/(LP1 + LP2) ratio in 0–20 cm soils of seven sites of Coochbehar and Malda.

	Malda				Coochbehar		
Depth	Site-1	Site-2	Site-3	Site-4	Site-5	Site-6	Site-7
0–5 cm	57.44	58.47	54.30	55.66	56.89	56.74	55.26
5–10 cm	53.88	60.82	56.68	57.08	55.76	53.72	55.93
10–20 cm	61.60	56.36	50.37	62.97	56.58	56.01	54.35

Significantly (*p*<0.05) higher RC fraction recorded in RM than RW system except in site-1 and site-7 where the RW dominated with higher values. The TOC of these two sites (site-1 and 7) studied from the main effect of cropping systems (Table 2) also showed the greater values in the RW system (10.24 and 12.40 g kg^-1^ under RW against 9.57 and 12.51 g kg^-1^ under RM systems in site-1 and site-7 respectively); these outcomes can explicate the variation of RC among the studied cropping systems. The sites of Malda showed higher concentrations of RC as compared to Coochbehar sites; because the soils of Malda are silt loam to silt clay in texture might be the strong reason behind stocking this fraction than in sandy soils (Coochbehar). Organic carbon in the fine silt or clay fractions includes organo-clay complexes and mineral grains coated with organic matter represent passive soil organic carbon [49]. Interestingly, in sandy soils, we observed a maximum contribution of labile C fractions (LP1 & LP2) to TOC as compared to clayey soils of Malda (Fig 3) indicates the influence of soil texture on C decomposition. de Gerenyu et al. [50] quantified the different organic carbon pools like total, labile, and recalcitrant pools in former croplands of arable soil under winter wheat and land-use change from crops to permanent grassland showed that the abandonment of cultivated soils increased the recalcitrant SOC pool (20.6 g kg^-1^ in arable soil vs. 28.6 g kg^-1^ in 77-yr grassland). RC is a larger fraction and a slow turnover rate exists in the soil system [18]. In our study, the RC fraction was found as a major pool and it was contributed around 70–75% of TOC. Several researchers also reported that RC contributes a large amount of total C, i.e., 86% [20] and 98.9–99.6% [50].

RETRACTED

The stratification of C fractions in 0–20 cm soil depth was found to be greater in Malda than Coochbehar due to heavier soil texture in the former district than the latter. This showed that the distribution of TOC and its fractions was more proportionate in subsequent deeper layers (5–10 and 10–20 cm) of Coochbehar soils. Hence, the decrease in the amount of TOC with soil depth was much proportional in Coochbehar due to high sand content. Additionally, the moisture content in these soils was relatively higher than in Malda which allowed the labile C pools to move down the profile layers with the moisture. Moreover, high rainfall and lighter soil texture result in easier movement of hydrolysates in the soils of Coochbehar. Changes in C fractions were mostly noticed in the first top 3 cm soil depth and were diluted in the subsequent layer 0–18 cm depth [51]; such decrements in C fractions with soil depth is caused by a natural stratification by residue accumulation on the soil surface [41]. The slow decomposition of the residue on the surface in ZT results in a slower rate of incorporation, as a result, there will be an increase in surface accumulation of the SOC [52]. Consequently, stratification ratios varied accordingly and were strongly influenced by the soil texture. In the Coochbehar soils (sandy loam textured, recent alluvial Entisols), movement of TOC and its fractions may have occurred into the soil profile, resulting in lower stratification than that in the Malda soils of finer soil textured old alluvial Inceptisol. This result further corroborated from the correlation study; where we observed a positive relation of C fractions with clay particles in Malda and negative with sand indicated that these fractions were associated with clay which was more stable than in Coochbehar. The importance of clay can vary by region [53] but soil physical properties such as clay content and mineralogy control the C fractions in soil by influencing the susceptibility of soil C to microbial attack [21].

RETRACTED

## 5. Conclusions

Contrasting tillage and cropping systems under CASI practice resulted in a peculiar variation with respect to the soil types. Excess residue addition through the rice-maize system in conservation agriculture increased the soil sequestration of carbon specifically in upper layers due to slow decomposition, hence gradual attachment of the added organic matter helps in reducing the loss to the environment. The conventional system involved with tillage and residue incorporation improved the C fractions in lower soil depths. A strong correlation of C pools with TOC indicated that the C fractions may vary in definition and method of estimation but represent a portion of soil organic carbon with different turnover rates and are important in judging the soil quality. The novelty of this study is that revealing the importance of clay particles in enhancing the labile and recalcitrant C fractions in the soil system. We observed a strong association/stabilization of C fractions with clay in the old alluvial Inceptisol which showed a higher concentration of C fractions as compared to recent alluvial Entisol with coarse loam texture (high sand). However, the stratification study revealed that depth-wise distribution of TOC, LP1, LP2, and RC were higher in sandy soils due to its greater movement in the soil profile and an imbalance in the distribution of carbon was more prominent in clayey soils. Thus, C input through crop residues and their amount is much important for long-term C storage which is reflected in our study under the residue management practice as varied in different soil types.

## Supporting information

S1 Table Soil pH, total organic C, total N, texture, and bulk density (0–20 cm) of the experimental sites along with the profile description and taxonomic name. (DOCX)

S2 Table Interaction effect of tillage, cropping system, and soil depth on TOC (g kg^-1^) in different sites of Malda and Coochbehar. (DOCX)

S3 Table Interaction effect of tillage, cropping system, and soil depth on LP1 carbon (g kg^-1^) in different sites of Malda and Coochbehar. (DOCX)

S4 Table Interaction effect of tillage, cropping system, and soil depth on LP2 carbon (g kg^-1^) in different sites of Malda and Coochbehar. (DOCX)

S5 Table Interaction effect of tillage, cropping system, and soil depth on RC (g kg^-1^) in different sites of Malda and Coochbehar. (DOCX)
